# Four cases of cell cannibalism in highly malignant feline and canine tumors

**DOI:** 10.1186/s13000-015-0429-3

**Published:** 2015-11-02

**Authors:** Fernando Costa Ferreira, Maria João Soares, Sandra Carvalho, Liliana Borralho, Gonçalo Vicente, Sandra Branco, Jorge Correia, Maria Conceição Peleteiro

**Affiliations:** CIISA, Interdisciplinary Centre of Research in Animal Health, Faculdade de Medicina Veterinária, Universidade de Lisboa, Av. da Universidade Técnica, 1300-477 Lisbon, Portugal; Clinica Veterinária do Oriente, Rua Nova dos Mercadores, 13 R/C Dto. 1990-176, Lisboa, Portugal; Veterinary Teaching Hospital, Faculty of Veterinary Medicine, Universidade de Lisboa, Av. da Universidade Técnica, 1300-477 Lisboa, Portugal; ICAAM - Institute for Mediterranean Agrarian and Environmental Sciences, University of Evora, Mitra, Ap. 94, 7006-554 Evora, Portugal

**Keywords:** Cell cannibalism, Neoplasia, Carcinoma, Mesothelioma, Cytokeratin, E-cadherin

## Abstract

Four cases of tumors in which cell internalization was frequently visualized are reported: one feline mammary carcinoma, one feline cutaneous squamous cell carcinoma, one canine pulmonary squamous cell carcinoma and one canine pleural mesothelioma. Cell internalization was observed by cytology in two of these cases (the feline mammary tumour and the pleural effusion in the canine mesothelioma) and by histopathology in all but the canine mesothelioma. Immunohistochemical staining for pancytokeratin was positive for both internalized and host cells, while E-cadherin expression was frequently absent, although internalized cells occasionally stained positive. This cell-to-cell interaction seems to be associated with tumors displaying a strong epithelial-mesenchymal transitional phenotype, in which cancer cells become engulfed by other cancer cells. Such event could be regarded as an important hallmark of very high malignancy.

## Background

Cell-to-cell interaction is a common phenomenon reported in inflammatory tissues, where macrophages engulf dying neutrophils and foreign material in a cooperative process during inflammatory/infectious diseases [1]. So far, three different mechanisms of cell-to-cell interaction have been described involving tumor cells: cannibalism, emperipolesis and entosis [2]. Briefly, cannibalism is the active internalization and destruction of dead or living tumor cells by other engulfing cells; emperipolesis is the phagocytosis of intact hematopoietic cells, mainly neutrophils, lymphocytes and plasma cells by host cancer cells; and entosis is a mechanism of homogenous live-cell invasion resembling a parasite-cell interaction, such that the invading cell seems to take the initiative in being internalized [2]. Recent studies have proven that these mechanisms have different cell recognition and cell penetration strategies [3–5]. However, there is much speculation around the possible benefits of such cell internalization events to either tumor or host.

In this study, the authors describe and discuss four cases of highly malignant tumors in which cell internalization was a frequent phenomenon. To the best of our knowledge, these internalization mechanisms have not been considered relevant in establishing diagnosis or prognosis in veterinary oncology.

## Case presentations

### Feline cases

#### Case one

A 9-year-old spayed European shorthair female cat was euthanized at the owner’s request, after a two-month history of a rapidly growing right inguinal mammary carcinoma diagnosed by cytology. At necropsy, a 4 cm nodule was present in the right inguinal mammary gland, along with several metastatic nodules identified in lymph nodes, lungs and in various muscles. Tissue samples were processed as usual for routine microscopical observation.

Histology of the mammary tumor revealed neoplastic cells arranged in nests within lobules. Extensive areas of necrosis were present and, in small and rare fields, tubular differentiation could be seen. The neoplastic cells were round or pleomorphic, measuring between 10 and 50 μm in diameter. The nuclei were either vesicular or hyperchromatic, occasionally deformed. Mitoses were frequent (8–10 dividing cells per ten high power fields). The lymphatic vessels in the periphery of the tumor were packed with neoplastic cells. In some areas, cancer cells appeared enlarged with a deformed, signet-ring nucleus due to the intracytoplasmic presence of an internalized cell similar to its host, albeit smaller, surrounded by a vacuole (Fig. 1a). The nuclei of the internalized cells were either normal or picnotic. Cellular internalization of tumor cells was similarly identified in the lung metastasis. The mammary tumor was diagnosed as a highly malignant metastatic solid carcinoma, exhibiting images of cell internalization. The re-evaluation of cytology smears cells revealed examples of the same type of cell internalization (Fig. 1b).

**Fig. 1:** Case 1. Solid mammary carcinoma. Cat. **a** – A small number of round tumor cells can be seen containing other tumor cells within a vacuole (arrows), giving the enclosing cell a signet ring-like appearance (HE). **b** – Cytology smear of the tumor in which a cell can be seen engulfing another (arrow) (Giemsa). **c** - IHC, anti-pancytokeratin antibody. Tumor cells stain positive, including internalized cells, one to the left and two to the right of the image. Mayer’s hematoxylin counterstain. **d** - IHC, anti-E-cadherin. Tumor cells show either homogenous cytoplasmic staining (lower arrow) or are almost completely negative (upper arrow) in contrast with the positive membrane staining of the surrounding tumor cells. Mayer’s hematoxylin counterstain

To confirm the epithelial nature of internalized cells and evaluate the presence of cell-adhesion molecules between outer and inner cells, immunohistochemistry for pancytokeratin and E-cadherin were performed, following the protocols described in Table 1. As expected, tumor cells, as well as their internalized targets, exhibited strong cytoplasmic staining for pancytokeratin (Fig. 1c). Cannibalizing cells showed positive membrane and/or diffuse cytoplasmic staining for E-cadherin, while internalized cells were only occasionally positive (Fig. 1d).

**Table 1:** Antibodies used and technique details

Antigen	Clone/Source	Retrieval	Dilution, incubation time	Detection system/Source
Pancytokeratin	Clone AE1/AE3 (DAKO)	Microwave 900W 5 min + 600W 15 min (Tris EDTA pH 9.0, Novocastra™ Epitope Retrieval Solution, Leica Biosystems, Wetzlar, Germany	1:100 60min RT	Novolink (Leica Biosystems)
Vimentin	Clone V9 (DAKO)	Microwave 900W 15 min (Tris EDTA pH 9.0, Novocastra™ Epitope Retrieval Solution, Leica Biosystems, Wetzlar, Germany)	1:50 60 min RT	Novolink (Leica Biosystems)
E-cadherin	Clone 36 (Ventana, Tucson, USA)	Microwave 600W 15 min (citrate buffer pH 6.0)	Ready to Use 60 min RT	Novolink (Leica Biosystems)

### Case two

A 15-year-old female cat was presented for consultation due to a large ulcerated mass in the upper abdominal region which was surgically removed. The tumor measured 9x6x3cm and was submitted to histological processing for routine microscopic observation. Histology revealed proliferation of keratinized epithelial cells organized in lobules, anastomosing cords and aggregates that frequently remained connected to the epidermis. Neoplastic cells were pleomorphic, varying from 50 to 120 μm in diameter. The mitotic index was high, with six dividing cells per ten high power fields. Images of cell internalization similar to the ones described in the first case were very frequent (Fig. 2a). The diagnosis was of highly infiltrative squamous cell carcinoma with lymphatic invasion, exhibiting images of cell internalization.

**Fig. 2:** Case 2. Squamous cell carcinoma. Skin. Cat. **a** & **b** – Images of cell internalization can be seen on the left and right in A, and in the centre in B, showing the signet-like appearance of the cannibal cells (HE). **c** - IHC, anti-pancytokeratin antibody. Two positive tumor cells can be seen. Mayer’s hematoxylin counterstain. **d** - IHC, anti-E-cadherin. Cannibalized tumor cells may be negative (lower arrow) or exhibit membrane staining (upper arrow). Tumor cells show positive cytoplasmic and membrane staining. Mayer’s hematoxylin counterstain

Immunohistochemical staining for pancytokeratin and E-cadherin were again performed as described in case one. Both tumor and internalized cells exhibited a strong cytoplasmic staining for pancytokeratin (Fig. 2c), while only cannibalizing cells consistently stained positively for E-cadherin. Internalized cells only occasionally stained for this marker (Fig. 2d).

The cat was euthanized at the owner’s request one month after surgery, due to severe ulceration of the skin in the area were the tumor was first removed, with no response to therapy.

### Canine cases

#### Case three

A 12-year-old intact male Labrador was euthanized after marked deterioration of its clinical condition following swelling and pain in the right hind leg with no response to treatment. Necropsy revealed a 3 cm nodule in the right posterior pulmonary lobe. Tissue samples were collected and processed as usual for routine microscopical observation. Histology revealed that the pulmonary nodule corresponded to a pleomorphic tumor consisting of lobules of compact spindle to polyhedral cells with occasional central abrupt keratinization. Necrosis was extensive. Mitoses were rare (1–2 dividing cells per ten high power fields). In the periphery of the nodule, alveoli were filled with numerous large round cells, 26 to 54 μm in diameter, revealing very frequent images of cell internalization, similar to the ones described in cases one and two (Fig. 3a). Fibrosis of the alveolar septa was very marked in these areas. Metastases of the lung tumor were identified in the right leg muscles, kidneys, left adrenal gland and right testicle. Cell internalization was not evident in the metastases. The diagnosis was of metastatic poorly differentiated squamous cell carcinoma of the lung with large areas of spindle-cell variant, exhibiting images of cell internalization.

**Fig. 3:** Case 3. Squamous cell carcinoma. Lung. Dog. **a** - Alveoli in the periphery of the tumor are filled with numerous round cells, with very frequent images of cell internalization (arrows) (HE). **b** - IHC, anti-pancytokeratin antibody. Tumor cells are positive (internalized cells included - two on the left and one on the right). Mayer’s hematoxylin counterstain

To confirm the epithelial nature of internalized cells, immunohistochemistry for pancytokeratin was performed according to the protocol described in Table 1. Tumor cells exhibited a strong cytoplasmic staining for pancytokeratin, along with the internalized cells (Fig. 3b).

### Case four

An 11-year-old intact female Boxer was presented with a severe pleural effusion (1500 mL). The cytological diagnosis of the effusion was of neoplasia with pleural dissemination with no clear distinction between carcinoma and mesothelioma. Frequent images of cellular internalization were present in the smears (Fig. 4a). The dog started chemotherapy with intrathoracic carboplatin but the pleural effusion persisted. Four weeks after the first presentation the dog was euthanized at the owner’s request. Upon necropsy, a large mediastinal mass (11x4x4 cm) was identified as well as various small nodules dispersed throughout the parietal pleura and diaphragm (Fig. 4b). Tissue samples were collected and treated for routine histological processing. Histology of the mediastinal mass revealed a poorly demarcated neoplasia infiltrating the adipose tissue displaying extensive areas of necrosis. The tumor organization involved two different types of tissues (Fig. 3c) with loosely arranged cells suggesting a sarcomatoid neoplasia and others of epithelial nature with cells organized in single layers covering papillary infoldings into cystic spaces filled with acidophilic content. Tumor tissue in the small nodules in the parietal pleura and diaphragm was mostly formed by lobules of loosely arranged sarcomatoid cells. The diagnosis was of pleural multicystic biphasic mesothelioma disseminated through the pleural cavity with severe pleural effusion showing frequent images of cell internalization.

**Fig. 4:** Case 4. Mesothelioma. Pleural cavity. Dog. **a** - Pleural effusion cytology smear showing frequent images of cellular internalization (arrows) (Giemsa). **b** – Large mediastinal mass can be seen together with various small nodules dispersed throughout the parietal pleura (arrows). **c** – Part of the tumor (upper left) was organized in variably sized lobules limited by trabeculae of fibrous tissue, formed by loosely arranged cells almost devoid of cytoplasm, with round nuclei. Extensive necrosis is visible, possibly due to chemotherapy. In other areas (lower right) the tissue is organized in single layers of epithelial cells covering papillary infoldings into cystic spaces filled with acidophilic content. **d** - IHC, anti-pancytokeratin antibody. Only the cells of the epithelial component are positive. Mayer’s hematoxylin counterstain

Immunohistochemical labeling with pancytokeratin and vimentin was employed to confirm the diagnosis of mesothelioma (protocol available in Table 1). The sarcomatoid cells were positive for vimentin (Fig. 4c) and the epithelial cells positive for cytokeratin (Fig. 4d).

## Discussion

All tumors described here were diagnosed according to standardized classification criteria and were shown to be particularly aggressive. Indeed, all cases reported correspond to highly malignant categories within the tissues they affected: a solid carcinoma of the mammary gland [6], a squamous cell carcinoma of the skin [7, 8], a poorly differentiated squamous carcinoma of the lung [9] and a biphasic mesothelioma of the pleura [10]. Two of them (cases 1 and 2) showed lymphatic invasion and in two cases (1 and 3) strong metastatic potential was proven. In the first three cases, images of cell internalization were identified by histology of the primary tumors and also in the lung metastasis of case 1. Regarding mesothelioma in case 4, images of cell internalization were only found in the pleural effusion fluid. In fact, phagocytosis of dying tumor cells by human peritoneal mesothelial cells has been demonstrated [11], as well as cannibalism in malignant effusions, but this does not necessarily mean that cannibal cells were tumor cells themselves [12]. The large number of cannibal cells present in the pleural effusion could represent cell cannibalism of tumor cells by other tumor cells, or the phagocytosis of exfoliating tumor cells by mesothelial cells. Morphology and immunohistochemistry are not helpful in distinguishing normal from neoplastic mesothelial cells [13], Cell cannibalism as the internalization of cells by other cells was first reported in human malignant tumors over a century ago, having been described as a diagnostic marker of malignancy in cytology specimens [11]. The potent phagocytic activity of tumor cells has been referred to as a determinant of aggressive behavior in metastatic melanoma cells, with proteins such as ezrin being expressed on phagocytic vacuoles [14]. The internalized cells may remain alive for some time, but will eventually be digested by specific enzymes within a cannibalistic vacuole; the inhibition or down regulation of these enzymes seems to affect the phagocytic activity of tumor cells [3, 5]. It has been suggested that cannibal cells feed off the internalized cells, becoming particularly resistant to unfavorable conditions caused by low nutrient supply in quickly growing solid tumors [2].

The other described cell-in-cell event is emperipolesis, which affects hematopoietic cells, mainly lymphocytes that establish close connections with the target cell’s membrane that culminate in their internalization. Although emperipolesis has been described in human mammary tumors [15] and lymphoma [16], the fact that the internalized cells in the presented case were not lymphocytes, or any other type of hematopoietic cell, excludes this hypothesis. In fact, cytokeratin staining was detected in both internalized and engulfing cells, demonstrating their identical epithelial nature.

The less referred to cell-in-cell phenomenon is entosis, through which live epithelial tumor cells detach from the extracellular matrix and invade the neighboring cells, also of epithelial origin [2]. Live internalized cells may either be degraded by lysosomal enzymes or be released. The process has been described as a non-apoptotic cell death program driven by compaction force associated with adherens junction formation, representing an intrinsic tumor suppression mechanism for cells that are detached from the extracellular matrix [5]. This event was reported in pleural suspensions of human metastatic mammary tumor cells, showing negative staining for apoptotic markers, leading to the conclusion that the internalization process could be associated with entosis [11]. E-cadherin is the main member of the cadherin superfamily involved in epithelial cellular adhesion, and its altered expression has been related to poor differentiation and poor prognosis, in human and canine mammary tumors [17, 18]. In feline mammary metastatic tumors, the loss of both E-cadherin and β-catenin expression was shown to be more pronounced than in non-metastatic neoplasia [19]. Cells in culture were demonstrated to require adherens junctions to initiate entosis, the mechanism being directly linked to cell-cell compaction force in the absence of integrin [5]. In the cases reported here, the generally negative staining obtained for E-cadherin in internalized cells could be due to its altered expression, which would be in accordance with the strong malignant behavior of the tumor. However, no conclusion can be drawn as to whether such cells had functional adherens junctions prior to engulfment.

It may be easily accepted that, similarly to what is reported in humans, cell-in-cell events also take place in tumors in animals. To the best of the authors’ knowledge, these phenomena have been rarely described and valued in veterinary oncology. The only reference to the phenomenon is very recent report involving three cases of cell cannibalism of which only one is of homogenous internalization of cancer cells [20].

## Conclusions

The authors believe that the cell internalization phenomena in the presently described tumors could be qualified as cannibalism, as there is evidence of degradation of the internalized cells. Conversely, it could also be classified as entosis as this is a case of epithelial-in-epithelial cell internalization, eventually evading apoptosis. Clear distinction between both events is beyond the scope of the present work, and does not affect its prime objective: to draw the attention of pathologists to a characteristic that seems to be associated with tumors in which the epithelial-mesenchymal transition is very marked.

## Consent

Written informed consent was obtained from the animal owners' for the publication of this report and any accompanying images.
